# Application of Cement-Based Composite Nanomaterials in Prefabricated Thin-Wall Light Steel Structure Composite Wall

**DOI:** 10.1155/2022/6015826

**Published:** 2022-09-08

**Authors:** Xiaoxu Chen, Huatuo He, Lingzhao Huo, Zhaorong Chen

**Affiliations:** ^1^Faculty of Architectural Engineering, Guangdong Baiyun University, Guangzhou, Guangdong 510000, China; ^2^Sichuan Zhongyu Environmental Governance Co., Ltd., CITCI Envirotech, Guangzhou Co., Ltd., Guangzhou, Guangdong 510000, China; ^3^Guangzhou Country Garden Real Estate Co., Ltd., Guangzhou, Guangdong 510000, China; ^4^China Construction Fifth Engineering Bureau the Third Construction Co., Ltd., Changsha, Hunan 410004, China

## Abstract

In order to solve the problem of seismic performance of prefabricated concrete shear walls connected with ultra-high performance cement-based composite (UHPC) after short lap of steel bars, the author proposes a cement-based composite nanomaterial in the prefabricated thin-walled lightweight application in steel structure composite wall. In order to explore the influence of the axial compression ratio on its seismic performance, 1 is a cast-in-place shear wall with a design axial compression ratio of 0.2, and 3 is a prefabricated shear wall with a design axial compression ratio of 0.2, 0.33, and 0.47, respectively, all the specimens were mainly damaged by shear compression. The test results show that the cracking loads of specimens PW2 and PW3 are increased by 17.04% and 38.81%, respectively, the yield load is increased by 27.74% and 50.28%, respectively, and the peak load is increased by 25.29% and 48.4%, respectively. *Conclusion.* With the increase of the axial compression ratio, the crack resistance and bearing capacity of the specimens are significantly improved.

## 1. Introduction

The fabricated light steel composite structure refers to the light steel composite components composed of 0.8–10 mm thick cold-formed thin-walled steel or ordinary steel and concrete, structural plates and thermal insulation materials, shear wall, frame-shear wall, and frame-support structure are assembled by connecting structures such as beam-column and wall panel nodes, and using bolts, self-tapping screws or embedded parts and other fastening components [1]. The prefabricated light steel composite structure is mainly used in low-rise and multistorey buildings, and it is a prefabricated building structure system with good development prospects [2]. The prefabricated light steel composite structural components mainly include light steel composite columns, light steel composite beams, light steel composite floors, and light steel composite shear walls [3]. Light steel composite nonstructural components can be used as peripheral retaining walls, partition walls, etc., and are suitable for low-rise, multistorey, and high-rise buildings [4]. The light steel composite column mainly adopts the lightweight concrete-filled steel tubular column, and can also use the steel-reinforced concrete column and the square steel tube composite section column [5].

Typical light steel composite structures mainly include prefabricated cold-formed thin-walled steel structures, prefabricated light steel light concrete structures, layered prefabricated light steel frames-flexible support structures, and prefabricated light steel composite frames-light steel composite shear force wall structure [6]. (1) The prefabricated cold-formed thin-walled steel structure can be classified into modular prefabricated cold-formed thin-walled steel wall panel structure, panel-column structure, wall panel column structure, etc., that is, the structure is divided into column modules, wall modules, components such as composite floors and connectors, modules are prefabricated in the factory, and directly assembled and connected after being transported to the site; (2) The prefabricated light steel light concrete structure is based on the prefabricated light steel frame as the structural skeleton and industrial prefabricated structural system of cast-in-place light concrete; (3) “Flexible support” and “light steel composite shear wall” are the high-efficiency seismic units of the first line of defense, so the layered assembled light steel frame-flexible support structure and the assembled light steel composite frame-light steel composite shear wall structure is collectively referred to as fabricated light steel frame—high-efficiency seismic element structural system [7].

The main materials of the light steel light concrete structure are thin-walled lightweight steel, dismantling-free formwork, and new lightweight concrete, the light steel composite frame is formed by the combination of thin-walled light-steel and dismantling-free formwork, lightweight concrete is poured on the basis of the light steel composite frame to form a light steel light concrete wall without dismantling the formwork [8]. The feature of the structure is that the light steel frame and the light concrete work together, and the structural performance is good as shown in Figure 1.

## 2. Literature Review

The ultra-high performance cement-based composite material is a kind of compressive strength greater than 150 MPa obtained by conventional preparation technology, at the same time, it is an ideal new building material with good mechanical properties and durability [9]. It is well known that concrete materials have multiscale structural characteristics, and its microstructure affects the performance of the macrostructure [10]. Multiscale can be roughly divided into micro-scale, meso-scale, and macro-scale [11]. On the microscopic scale, the cement hydration product provides the gelling ability and constitutes the microstructure of the concrete material. On the microscopic scale, the cement and sand constitute the cement mortar, and the cemented stone constitutes the concrete material. On the macro-scale, stones and cement mortar form concrete materials, which harden into various concrete components and structures [12]. Throughout the research on the antiexplosion performance of concrete, it is mainly based on macroscopic structural design and other aspects, as a typical heterogeneous composite material, concrete, considering its multiscale characteristics, at the same time, the performance analysis and structural design are carried out from the microscopic, mesoscopic, and macroscopic scales to better improve the antiknock and impact resistance of cement-based composites [13]. Cement-based composite materials refer to materials with new properties obtained by combining the hardened cement paste formed by the hydration and hardening of cement and water as the matrix and other various inorganic, organic, and metal materials; during the coagulation and hardening process of this material, phenomena such as dry shrinkage and bleeding will occur, which lead to the random existence of a large number of micropores and interface cracks and other defects in the material [14].

The connection method is one of the most important factors affecting the seismic performance of the fabricated structure, the traditional connection methods mainly include direct lap connection, grout anchor connection, and sleeve grouting connection [15]. Due to the relatively long lap length of the steel bar and more wet operations on-site, the direct lap joint has no significant application advantages in prefabricated buildings. Grout anchor connection and sleeve grouting connection have high requirements on construction accuracy, the connection of steel bars is difficult, and the quality of grouting is not easy to detect [16].

Ultra-high performance cementitious composites (UHPC) have excellent mechanical properties such as high strength, high toughness, self-compacting, and low porosity [17]. Some scholars applied UHPC to the prefabricated concrete frame structure, invented the high-efficiency connection technology of UHPC after the short lap of the steel bar, and conducted the pull-out test on 15 central specimens, the test results show that the critical anchorage length of steel bars and UHPC is 4d (d is the diameter of steel bars), in addition, the quasi-static test results of beams, columns, frame edge nodes and two-story two-span frames show that, when the lap length of the steel bar is 10d, the fabricated member using this connection technology, its seismic performance is basically equivalent to that of all cast-in-place members [18]. On this basis, it is further proposed that the precast concrete shear wall is connected with the reinforced straight anchor short lapped (10d) post-cast UHPC through the low-cycle repeated load test to test its seismic performance such as bearing capacity, hysteretic energy dissipation, displacement ductility, stiffness, and strength degradation [19].

## 3. Methods

### 3.1. Specimen Design and Production

A total of 4 shear wall specimens were designed and fabricated in the test, of which the specimen SW1 was a cast-in-place specimen, the design axial compression ratio was 0.2, and the design axial compression ratio was calculated according to formula (1). Specimens PW1, PW2, and PW3 are prefabricated specimens, and the design axial compression ratios are 0.2, 0.33, and 0.47, respectively.

(1) $$\begin{array}{c} n=1.2\times \frac{N}{f_{c}A}. \end{array}$$

In the formula: *n* is the design axial pressure ratio; *N* is the applied vertical axial pressure; *f*_c_ is the design value of the concrete compressive strength; and A is the cross-sectional area of the shear wall.

The geometric dimensions and reinforcement of each specimen are the same, and they are all composed of ground beams, walls, and top loading beams [20]. Referring to the research of relevant experts and scholars and comprehensively considering the laboratory site conditions and the bearing capacity of the loading device, the wall thickness of each specimen is taken as the minimum value of 160 mm, the wall height is 2800 mm, and the wall width is taken as 1300 mm according to 8 times the wall thickness, dark columns are set within 200 mm of both ends. All steel bars are HRB400 grade steel bars, the vertical bars of the hidden column are 4Φ16, the stirrups of the hidden column are Φ8@150, and a stirrup with a diameter of 8 is set in the UHPC postcasting section of the hidden column. The vertical distribution rib is 8Φ8@180/200; the horizontal distribution rib is Φ8@150.

When making the specimen, the ground beam was poured first, and the wall and the loading beam were poured at the same time, after the prefabricated wall was hoisted, the mold was sealed and UHPC was poured, the top surface of the ground beam and the bottom of the prefabricated wall were rough surfaces. The UHPC postcasting section is reserved at the bottom of the prefabricated specimen wall, the height of the postcasting section is 180 mm for the dark column, and 100 mm for the middle of the wall. The lap length of the vertical steel bars in the postcasting section: the vertical steel bars of the dark column are 160 mm, and the vertical distribution bars in the wall are 80 mm. In order to facilitate hoisting, outriggers are set in the postcast section at the bottom of the prefabricated shear wall, the width of the outriggers is 100 mm and the thickness is 100 mm, that is, a channel with a thickness of 60 mm is reserved so that UHPC can circulate between the dark column and the inner wall.

### 3.2. Material Properties

The specimens were made of C40 concrete, and the UHPC was made of ultra-high performance concrete, the distribution ratio of each component of UHPC is shown in Table 1. A standard cube test block was reserved when the test piece was made, and was cured under the same conditions as the test piece, the measured compressive strengths of concrete and UHPC standard cubes were 46. 0MPa and 110MPa, respectively. The measured yield strength *f*_y_, yield strain *ℰ*_y_, tensile strength *f*_*u*_, and elongation *δ* of the steel bar properties of each diameter are shown in Table 2. When calculating the yield strain of steel bars, the elastic modulus is taken as *E*_s_=2.0 × 10^5^MPa.

### 3.3. Test Loading

This test is carried out in the structural laboratory, and the specimen is fixed on the laboratory reaction foundation by two ground anchor bolts. The designed axial pressure ratio of specimen SW1 and specimen PW1 is 0.2, calculated according to formula (1) and rounded up, and the applied axial pressure is 660 kN. The design axial pressure ratios of the specimens PW2 and PW3 are 0.33 and 0.47, respectively, and the applied axial pressures are 1100 and 1560 kN, respectively. The vertical load is applied by a 2000 kN hydraulic jack, there is a two-way pulley on the top of the jack.

The horizontal load is controlled by a mixture of load and displacement, during the test, the load corresponding to the first yield of the longitudinal reinforcement of the dark column is the nominal yield load, and the corresponding displacement is the nominal yield displacement Δ_*q*_, load control is adopted before the specimen yields, and each load cycle is performed once, and the increment is 40 kN. Displacement control was adopted after the specimen yielded, and the displacement was cycled 3 times for each stage, and the increment was an integer multiple of Δ_*q*_, until the load dropped to 85% of the peak load, or the test was terminated when the specimen showed obvious failure. *P*_*y*_ is the load peak value corresponding to the load control loading.

### 3.4. Measurement Content and Measurement Point Arrangement

The main contents of the test measurement are: vertical load, horizontal load, horizontal displacement, vertical steel bar strain, etc. The vertical load and horizontal load are collected by the hydraulic loading system with its own force sensor. The horizontal displacement of the vertex is collected by arranging the cable displacement meter at the center of the end section of the loading beam, the displacement of the wall at different heights is collected by arranging the rod displacement meter at the corresponding position of the central axis of the wall. The vertical steel bar strain is collected by pasting steel bar strain gauges: the specimen SW1 is arranged with a strain gauge 20 mm below the top surface of the ground beam, and the specimen is placed 20 mm below the top surface of the ground beam, and strain gauges are arranged 20 mm above the interface of the postcasting section at the bottom of the wall. In order to monitor the displacement of the ground beam, tie rod displacement gauges are arranged at the two ends, the top surface and the two sides of the ground beam diagonally.

### 3.5. Test Phenomenon

#### 3.5.1. Specimen

When the horizontal load reaches 160 kN, the first horizontal fine crack appears at the wall end about 170 mm from the top surface of the ground beam, which is defined as the cracking load. When loaded continuously, the horizontal cracks are extended, and new horizontal cracks appear one after another within 1/3 of the wall height at the bottom of the wall. When the load reaches ±200 kN (the horizontal loading stipulates that pushing is positive and pulling is negative), small cracks appear on the connection surface between the bottom of the wall and the ground beam. The existing horizontal cracks begin to develop obliquely downward. When the load reaches −240 kN, the bottom of the wall and the crack of the ground beam are connected to form a through-crack, and some of the oblique cracks extend beyond the middle of the wall to form a cross oblique crack. When the load reaches −260 kN, the vertical steel bars of the dark column yield successively, at this time, the maximum crack width is 0.37 mm, and the horizontal displacement of the vertex is 14.56 mm. The next level is changed to displacement control loading, and the control loading displacement is an integer multiple of 15 mm.

When the horizontal displacement of the vertex reaches 30 mm, the cracks on the connection surface between the wall and the ground beam increase significantly, and the corner of the tension side is lifted by about 3 mm. The corners of the side walls under pressure are compressed and split. When the horizontal displacement reaches ±45 mm (the horizontal displacement is defined as positive for pushing and negative for pulling), the concrete of the dark columns at both ends will be crushed and peeled off. When the horizontal displacement of the apex reaches ±80 mm, the concrete of the dark column is crushed, the steel bar buckles the outer drum, and the specimen is obviously damaged, for the safety of the test, the loading is stopped.

#### 3.5.2. Specimen PW1

When the horizontal loading reaches −180 kN, a horizontal crack with a length of about 300 mm appears within the range of 20–30 mm upward from the junction surface of the postcast section of the dark column, and this level of load is defined as the cracking load. Continuing to load, multiple horizontal cracks appeared one after another in the height range of 200–1200 mm from the bottom to the top of the wall, and multiple through horizontal cracks appeared on the side of the wall. When the horizontal loading reaches ±220 kN, the original horizontal cracks begin to develop obliquely downward. When loaded to −240 kN, a tiny crack appeared on the connection surface between the wall and the ground beam. Within the range of 400–800 mm from the top surface of the ground beam, there are two oblique cracks extending beyond the middle of the wall, forming crossed oblique cracks. When the load reaches 280 kN, the cracks between the wall and the ground beam pass through. When loaded to ±300 kN, the vertical steel bar of the dark column yields in tension, the maximum crack width is 0.32 mm, and the horizontal displacement of the vertex is 17.64 mm. The next stage starts to control the loading by displacement, in order to compare with the specimen, the control loading displacement is an integer multiple of 15 mm.

When the horizontal displacement of the apex reaches 30 mm, the cracks on the connection surface between the wall and the ground beam increase significantly, and the corners on the tension side tend to be slightly lifted. The horizontal through-cracks above the interface between UHPC and concrete on the wall side increased, and the maximum crack width was 3.05 mm. No cracks appeared in the postcasting section of UHPC. Continuing to load, the existing cracks grow and extend, and no new cracks appear. When the horizontal displacement of the apex reaches ±75 mm, the steel bar above the UHPC postcasting section of the left hidden column is buckled and the concrete is crushed and peeled off, the bearing capacity of the specimen has dropped to 85% of the peak load, and the loading is stopped.

#### 3.5.3. Specimen PW2

When the horizontal loading reaches 200 kN, the first horizontal crack appears above the interface between the UHPC and the concrete. Continuing to load, multiple horizontal cracks appear on the wall within 1200 mm from bottom to top, the side of the crack penetrates and extends to the front for about 150–200 mm. When the load reaches 280 kN, through-cracks appear at the connection between the wall side and the ground beam, and extend to the front for about 100 mm. Two existing horizontal cracks developed obliquely downward within the height range of 800–1000 mm from the bottom to the top of the wall, with a length of about 560 mm. When the load reaches ±340 kN, a through-crack is formed at the connection between the bottom of the wall and the ground beam, the vertical reinforcement yields, and the maximum width of the crack is 0.36 mm, at this time, the horizontal displacement is 13.81 mm. The next stage starts to load with displacement control, and the control loading displacement is an integer multiple of 14 mm.

When the horizontal displacement of the apex reaches 28 mm, two vertical cracks about 50 mm long and two oblique cracks about 70 mm long appear in the UHPC at the bottom of the dark column on the tension side. When the horizontal displacement reaches ±42 mm, the concrete above the interface between the UHPC and the concrete of the two ends of the concealed column is slightly pressed and peeled off, and the tension side of the end of the concealed column is lifted by about 5–6 mm. An existing oblique fissure at the bottom of the dark column on the left enlarged and extended, forming a main oblique fissure penetrating the dark column and developing to the side. When the horizontal displacement increases to ±56 mm, the bearing capacity of the specimen dropped to 85% of the peak load under positive loading, but the bearing capacity of the specimen still increases under negative loading. When the horizontal displacement of the vertex increases to −80 mm, the negative bearing capacity of the specimen dropped to 85% of the peak load, and the loading is stopped.

#### 3.5.4. Specimen PW3

When the horizontal loading reaches 240 kN, a horizontal crack appears on the interface between the UHPC of the dark column and the concrete. When the load reaches −260 kN, the second horizontal crack appears at about 20–30 mm above the interface between the UHPC and the concrete, at the same time, a fine crack appeared at the connection between the UHPC and the ground beam on the side of the dark column, and it extended to the back of the wall for about 100 mm. When the load reaches ±360 kN, the existing horizontal cracks begin to develop obliquely downward. When the load reaches −400 kN, the vertical steel bar begins to yield, and the maximum crack width is 0.34 mm from the bottom to the top within the height range of 600 mm, and an oblique crack spans the middle of the wall. The cracks on the connecting surface between UHPC and the ground beam are not connected. At this time, the horizontal displacement of the vertex is −15.43 mm. The next stage starts to load with displacement control, and the control loading displacement is an integer multiple of 15 mm.

When the horizontal displacement of the apex is ±45 mm, the cracks in the connection surface between UHPC and ground beam increase obviously. There are many irregular cracks in the UHPC of the dark column at both ends, the maximum crack width of the connection surface between the UHPC of the dark column and the concrete is 1.72 mm, and the concrete above the connection surface is compressed. At this point, the wall cracks have been cleared, and no new cracks will appear if the loading continues. When the horizontal displacement reaches ±75 mm, the bearing capacity of the specimen dropped to 85% of the peak load, and the loading is stopped.

### 3.6. Destruction Form

The following conclusions are drawn from the analysis of the crack distribution and failure form of the four specimens:

1. On the whole, the cracks of each specimen are of bending-shear type, and the distribution state is relatively close. Each specimen is damaged by tensile yield of longitudinal reinforcement of edge members and crushed concrete, which is a typical shear compression failure.
2. When the axial compression ratio is the same, relative to the specimen, the failure zone of the specimen does not occur in the corner, but appears above the postcast section of the dark column, and there is no obvious damage in the postcast section of UHPC.
3. With the increase of the axial compression ratio, the distribution heights of the cracks in the specimens PW2 and PW3 decrease in turn, and the length of the horizontal section of the cracks decreases correspondingly, and the inclination of the inclined cracks increases. The cracking in the postcast section of UHPC is more obvious.
4. One side of the UHPC postcasting section of the PW2 concealed column of the test piece was severely damaged, while the other side was relatively intact, mainly due to the insufficient concrete protective layer due to the problem of the pouring quality, resulting in the failure of the reinforcement anchorage: the thickness of the concrete protective layer of the specimen is set to 15 mm, due to the construction deviation, the actual protective layer thickness of the damaged area is only 5 mm.

### 3.7. Hysteresis Curve

Specimen PW1 and specimen SW1 have similar hysteresis curves in shape, both of which are arcuate, with fuller hysteresis loops and better energy dissipation capacity. Before cracking, the surrounding area of the hysteresis loop of each specimen is very small, the curve is basically a straight line, and the specimen has no residual deformation and is in an elastic state. After yielding, the hysteresis loops of the specimens SW1 and PW1 are relatively stable, and the specimens have good deformation ability. Due to the accumulation of concrete plastic damage, the stiffness of the specimens SW1 and PW1 gradually deteriorated, and a slight pinching phenomenon appeared in the center of the hysteresis curve. The hysteresis curves of specimen PW2 and PW3 are similar in shape, and both are inverse S-shape. Compared with the increase of the axial compression ratio of the specimen PW1, the surrounding area of the hysteresis loop of the specimen PW2 and the specimen PW3 decreased, the pinching phenomenon was more obvious, and the energy dissipation capacity of the specimen decreased.

### 3.8. Stiffness Degradation

The stiffness of the specimen can be characterized by the loop stiffness, and its expression is

(2) $$\begin{array}{c} K_{i}=\frac{\sum_{j=1}^{n}F_{ij,\max}}{\sum_{j=1}^{n}\Delta_{ij}}. \end{array}$$

In the formula: *K*_*i*_ is the load ring stiffness of the *i*-th level; *F*_*ij*,max_ is the *i*-th level loading and the *j*th level maximum cyclic load; Δ_*ij*_ is the displacement corresponding to *F*_*ij*, max _.

### 3.9. Strength Degradation

The intensity degradation can be characterized by the intensity degradation coefficient *λ*, which is expressed as

(3) $$\begin{array}{c} \lambda_{j}=\frac{F_{i}^{j}}{F_{i}^{j-1}}. \end{array}$$

In the formula, *λ*_*i*_ is the strength degradation coefficient of the *j*th cycle; *F*_*i*_^*j*^  is the *i*-th level load, the peak load of the *j*th cycle.

### 3.10. Energy Consumption Capacity

The energy dissipation capacity of the specimen can be measured by the equivalent viscous damping coefficient *h*_*e*_, and its expression is

(4) $$\begin{array}{c} h_{e}=\frac{1}{2\pi }\frac{S_{\text{DAB}}+S_{\text{BCD}}}{S_{\Delta \text{OAN}}+S_{\Delta \text{OCM}}}, \end{array}$$

where *h*_e_ is the equivalent viscous damping coefficient; *S*_DAB_+*S*_BCD_ is the area enclosed by the hysteresis loop. *S*_△OAN_ and *S*_△OCM_  are the areas of △OAN and △OCM, respectively.

## 4. Results and Analysis

The skeleton curve of each specimen is shown in Figure 2. Among them, the first crack in the specimen is regarded as the cracking state, and the yield load and yield displacement are determined by the energy equivalent method. The maximum load of the skeleton curve is taken as the peak load, and the corresponding displacement is the peak displacement. The limit state is taken as the bearing capacity of the specimen which drops to 85% of the peak load. Compared with specimen SW1, the cracking load, yield load, and peak load of specimen PW1 were increased by 12.36%, 4.34%, and 7.56%, respectively. After the peak load, the skeleton curves of the specimens PW1 and SW1 are relatively gentle, the bearing capacity decreases slowly, and the specimens have good ductility and deformation capacity. The larger the axial compression ratio, the larger the slope of the skeleton curve in the elastic stage, which means that with the increase of the axial compression ratio, the initial stiffness of the shear wall increases accordingly. Compared with the specimen, the specimen and cracking loads are increased by 17.04% and 38.81%, respectively, the yield load is increased by 27.74% and 50.28%, respectively, and the peak load is increased by 25.29% and 48.4%, respectively, it shows that with the increase of the axial compression ratio, the crack resistance and bearing capacity of the specimens are significantly improved. When the axial compression ratio increases, the yield displacement of the specimen does not change much, but the peak displacement and limit displacement decrease accordingly. After passing the peak point, the descending section of the curve is steeper, indicating that the larger the axial compression ratio, the worse the ductility and deformation capacity of the shear wall, and the faster the strength degradation.

The stiffness degradation curve of each specimen is shown in Figure 3, from Figure 3, it can be seen that the stiffness degradation curve of each specimen is basically the same: the stiffness degradation was fast at the initial stage of loading, and the stiffness degradation speed was slow after yielding. With the increase of displacement and the development of cracks, the ring stiffness of each specimen tended to the same level. The stiffness degradation curve of the specimen PW1 basically coincides with that of the specimen SW1, and the loop stiffness of the specimen PW1 is slightly larger than that of the specimen SW1. With the increase of the axial compression ratio, the ring stiffness of the specimen increases correspondingly at the same displacement, the main reason is that the increase of the axial compression ratio inhibits the development of cracks and the increase of deformation, it shows that the increase of the axial compression ratio can improve the lateral displacement resistance of the shear wall.

1. In general, the strength degradation coefficient of the third cycle of each specimen is greater than that of the second cycle, indicating that with the increase of the number of loading cycles, the strength degradation of the specimen slows down.
2. For the same specimen, with the increase of the displacement amplitude, its strength degradation coefficient decreases slowly, indicating that the strength degradation rate of the specimen is relatively stable as the displacement increases. The strength degradation curve of the specimen PW2 under forward loading has obvious bends, mainly because the UHPC protective layer of the hidden column is insufficient, which leads to the failure of the vertical reinforcement of the left hidden column, resulting in a rapid decrease in the bearing capacity. A similar phenomenon also appeared when the specimen PW3 was negatively loaded.
3. When the specimen SW1 is 1 times the yield displacement amplitude, the strength degradation coefficient is greater than 1, this is because the horizontal displacement of the apex in the second cycle is greater than the horizontal displacement of the apex in the first cycle, this lead to increased load. Besides, the trend of the strength degradation coefficient curve is not much different from that of the specimen PW1, which indicates that the prefabricated specimen has better bonding and anchoring performance of steel bars and is basically equivalent to the cast-in-place specimen.
4. The trend and numerical value of the strength degradation coefficient of the specimens PW2 and PW3 are not much different from those of the specimen PW1 in general, indicating that the reinforcement and UHPC can still be reliably bonded and effectively transmitted by increasing the axial compression ratio.

The equivalent viscous damping coefficient-vertical horizontal displacement relationship curve of each specimen is shown in Figure 4. It can be seen from Figure 4 that

1. The trend of the equivalent viscous damping coefficient curve of each specimen is roughly that the equivalent viscous damping coefficient decreases with the increase of the load, and the equivalent viscous damping coefficient increases with the increase of the displacement after yielding. The main reasons are: before yielding, the bearing capacity of the specimen increases sharply with the increase of the load, but the displacement is small, the hysteresis loop is narrow, and the performance of the steel bar is not fully exerted. After yielding, the bearing capacity of the specimen increases slowly, but the displacement increases rapidly, the hysteresis loop is fuller, the performance of the steel bar is fully exerted, and the energy consumption of the specimen is better.
2. Before yielding, the PW1 equivalent viscous damping coefficient curve of the specimen basically coincides with that of the specimen. After yielding, the curves of the equivalent viscous damping coefficients of the two specimens are similar, indicating that the prefabricated specimens have similar energy dissipation capacity as the cast-in-place specimens.

## 5. Conclusion

The author proposes the application of cement-based composite nanomaterials in prefabricated thin-walled light steel structure composite walls, on the whole, the cracks of each specimen are of bending-shear type, and the distribution patterns are relatively close. For each specimen, the longitudinal reinforcement of the edge members and the corresponding beam reinforcement yielded in tension, and the concrete was crushed and finally destroyed, which was a typical shear compression failure. When the axial compression ratio is the same, compared with the cast-in-place specimen, the crack resistance, bearing capacity and stiffness of the prefabricated specimen are improved, and the ductility and energy dissipation capacity are similar. With the increase of the axial compression ratio, the crack resistance, bearing capacity, and stiffness of the specimens are significantly improved, while the ductility and energy dissipation capacity are decreased. The prefabricated concrete shear wall structure with UHPC cast after the short lap of the steel bar straight anchor has good anchorage performance and can effectively transmit force, which is equivalent to the requirement of full cast-in-place.

## Figures and Tables

**Figure 1:** Cement-based composite nanomaterials.

**Figure 2:** Skeleton curve of each specimen.

**Figure 3:** Stiffness degradation curve of each specimen.

**Figure 4:** Equivalent viscous damping coefficient-vertical horizontal displacement curve of each specimen.

**Table 1:** Distribution ratio of each group of UHPC.

Component	Superfine cement	Silica fume	Quartz sand	Finely ground filler	Superplasticizer	Water	Super fine steel fiber
Proportion	1.0	0.3	1.34	0.3	0.005	0.2	0.02

**Table 2:** Mechanical properties of steel bars.

Specification	*f*_y_/MPa	*ε*_y_/(×10^−6^)	*f*_u_/MPa	*δ*/%
Φ8	525.94	2 630	701.25	23.13
Φ16	557.66	2 788	698.76	21.46

## Data Availability

The data used to support the findings of this study are available from the corresponding author upon request.
